The article "Spread of Online Public Opinion of Animal Epidemic Emergency: A Case Study of the H7N9 Incident Based on Healthcare Data Analytics" was retracted in 2022. Reason: concerns about the peer review.

# Spread of Online Public Opinion of Animal Epidemic Emergency: A Case Study of the H7N9 Incident Based on Healthcare Data Analytics

**DOI:** 10.1155/2021/1512742

**Published:** 2021-11-30

**Authors:** Yanling Li, Xianyi Shen

**Affiliations:** College of Public Administration and Law, Hunan Agricultural University, Changsha, China

## Abstract

Qualitative and quantitative analysis of online public opinion of the H7N9 animal epidemic incident in 2013 were conducted based on social network analysis (SNA) theories, SNA method, and life cycle theories. Trend and features of evolution of online public opinion of animal epidemic emergency were explored and structural characteristics of key nodes in these public opinion spreading networks were identified. The stages of spreading of public opinion of animal epidemics were investigated. This study provides references for the government to cope with online public opinion of animal epidemic emergencies in the future.

## 1. Introduction

Recently, animal epidemic emergencies have been a severe issue globally. Animal epidemic emergencies not only affect the development of national livestock industry but also endanger the lives of people. With the rapid development of the Internet and the popularization of media platforms, the public can obtain information of animal epidemic emergencies through multiple channels, which poses a challenge to the government's emergency response to a certain extent [1]. Therefore, it is necessary to recognize and grasp the new features and rules of spreading of online public opinion of animal epidemic emergency and take active and effective measures to improve the ability to respond to online public opinion of animal epidemic emergency, which has become a topic worthy of high attention [2]. In this study, life cycle theory, social network analysis (SNA) theory, and SNA method were applied to the study of spreading of online public opinion of animal epidemic emergency. Firstly, the spreading of online public opinion of animal epidemic emergency was divided into three stages according to the life cycle theory, and the suggestions were provided to the government for the different stages, and then the public opinion spreading network of H7N9 animal epidemics was specifically targeted, which was analyzed by using the theory and method of social network. The key nodes in this network were identified and discussed. Finally, the evolution of online public opinion of animal epidemic emergency was revealed to provide theoretical and practical basis for the management of public opinion in such incidents in the future.

## 2. Online Public Opinion of Animal Epidemic Emergency and SNA

### 2.1. Online Public Opinion of Animal Epidemic Emergency

Online public opinion of animal epidemic emergency refers to the fact that netizens release animal epidemic emergency-based information on Weibo, SBS, and other cyberspaces, including emotions, attitudes, intentions, opinions, and behavioral tendencies [3], with the characteristics of suddenness, magnification, low ignition point, many contacts, and large impact [4]. Among the existing studies on the characteristics of life cycle of public opinion, scholars have proposed different online public opinion stage communication models: three-, four-, five- and six-stage communication models have been proposed through empirical evidence and analysis [5]. Initially, three-stage spreading model of online public opinion was proposed. Based on that, researchers have used individual cases as examples for empirical analysis and gradually proposed four-, five-, and six-stage communication models. The more general three-stage model is commonly used for empirical studies in conjunction with events. Cheng et al. adopted a three-stage model to divide the evolution of online public opinion into occurrence stage, outbreak stage, and gradual extinction stage. The “Yu Huan” case was analyzed in this way [6]. Gao et al. used a three-stage model to conduct an in-depth analysis of the online public opinion spreading of the Jiaduobao “barbecue” incident [7]. The naming of the three stages varies among academics; however, the connotation is basically the same. In the study of online public opinion spreading stage model, Zeng et al. concluded that the three-stage model was divided into three stages: occurrence, spreading, and integration [8].

The article "Spread of Online Public Opinion of Animal Epidemic Emergency: A Case Study of the H7N9 Incident Based on Healthcare Data Analytics" was retracted in 2022. Reason: concerns about the peer review.

In this paper, a three-stage model for the spreading of online public opinion of animal epidemic emergency process was adopted, including the occurrence stage, the spreading stage, and the fading stage (see Figure 1).

### 2.2. SNA

SNA is an analytical method to study the interrelationships between nodes in a particular environment, to uncover the characteristics of relationships, and to explore the impact of relationships on social structure [9]. Generally, SNA of online public opinion of animal epidemic emergency mainly covers network density, intermediate centrality, closeness centrality, core-periphery, out-in degree, and other structural measures. Herein, the H7N9 incident, which is a representative animal epidemic emergency, is selected for qualitative and quantitative analysis.

## 3. SNA of Spreading of Online Public Opinion of the H7N9 Incident

### 3.1. Stages of Spreading of the H7N9 Incident

This paper determines the development trend of the public opinion of the H7N9 incident based on the search index of keyword “H7N9” on Baidu index, as shown in Figure 2. The life cycle of online public opinion of the H7N9 incident consists of occurrence period, spreading period, and fading period (see Table 1).

The article "Spread of Online Public Opinion of Animal Epidemic Emergency: A Case Study of the H7N9 Incident Based on Healthcare Data Analytics" was retracted in 2022. Reason: concerns about the peer review.

### 3.2. Data Collection and Processing

The data used in this article to study the online public opinion of H7N9 animal epidemic emergency were collected from Sina Weibo through web crawlers and snowball sampling.

Firstly, the user nodes that initially posted “H7N9”-related information in microblog after the event were identified; secondly, a complete statistics of user nodes with high retweets were conducted; finally, 5 nodes (Toutiao News, Shanghai Morning Post, Sina Video, Beijing Evening, and MOP.com) were identified by random screening among the nodes that met these criteria.

After the initial nodes were determined, the retweet nodes and comment nodes under each tweet were counted, until there were no retweets or comments, and then all the reposting nodes were removed. Finally, a total of 2369 nodes were sorted out. Ucinet was used to establish an adjacency matrix to express the propagation relationship among nodes. The values of the edges of matrix were determined by combining the number of comments and the number of retweets of the nodes. The adjacency matrix was constructed by closely linking each node.  Figure 3 shows the overall online public opinion spread of the H7N9 incident. The structure and key nodes of the H7N9 incident public opinion spreading network were summarized and are shown in Figure 3. As observed, actors in key positions include Toutiao News, Hot topics in Weibo, and Kaifu Lee. Frequent interaction made it a key role in online communication.

### 3.3. Analysis of Network Density

The network density reflects the interaction degree of information spreading among netizens [12]. Assuming that the actual number of nodes in a directed network was *n*, then the maximum number of possible node connections was *n* (*n* − 1), and the directed network density (*D*) could be calculated:

(1) $$\begin{array}{c} D=\frac{n}{n\left(n-1\right)}. \end{array}$$

The measured network density of spreading of online public opinion of the H7N9 incident is shown in Table 2.

The public opinion spreading network of the H7N9 incident consisted of 2369 nodes and the actual number of interaction connection ties that occurred was 3178 (network density = 0.0005). Mayhew et al. used a random selection model to analyze the measurements to obtain a maximum density of network diagram of 0.5. In practical spreading of online public opinion, the number of connections of the complete graph was much larger than the number of connections of the actual graph [13]. The network density of public opinion spreading network was positively correlated with the interaction rate and connection between nodes. As observed, spreading of online public opinion of the H7N9 incident on Weibo showed loose actor connection, low overall network integrity, and low information interaction efficiency.

The article "Spread of Online Public Opinion of Animal Epidemic Emergency: A Case Study of the H7N9 Incident Based on Healthcare Data Analytics" was retracted in 2022. Reason: concerns about the peer review.

### 3.4. Analysis of Intermediate Centrality

The intermediate centrality reflects the mediating ability of a node, which is the ability of the node to occupy the shortest path between two other nodes. Hence, intermediate centrality is also known as “bridging” capability [14]. The higher the intermediate centrality of a node, the more resources and information it possesses, the more prominent the bridging ability, and the stronger the ability to control other actors. Therefore, it is also a key control node in spreading of online public opinion of animal epidemic emergency. The intermediate centrality (*C*_*B*_) was calculated as in (2). The shortest route number between node *j* and *k* containing node *n*_i_, *g*_*jk*_ (*n*_*i*_) was divided by the shortest route number between node *j* and node *k* (*g*_*jk*_).

(2) $$\begin{array}{c} C_{B}=\frac{\sum_{j<K}g_{jk}\left(n_{i}\right)}{g_{jk}}. \end{array}$$

The difference between the maximum intermediate centrality (*C*_*B*max_) in the network structure diagram and the intermediate centrality of a specific node (*C*_*Bi*_) was defined as the intermediate central potential. If the gap between the node and other nodes was larger, the intermediate central potential of the network was higher [15]. The intermediate central potential can be calculated by

(3) $$\begin{array}{c} C_{B}=\frac{2\sum_{i=1}^{N}\left(C_{B\max}-C_{Bi}\right)}{{\left(n-1\right)}^{2}\left(n-2\right)}. \end{array}$$

The measured intermediate centrality of spreading network of online public opinion of the H7N9 incident is shown in Table 3. As shown in Table 2, Toutiao News, a1400273289, Kaifu Lee, Changzhou Daily News Tongtong, Luo Yonghao Smartisan handphone, MOP.com, Cixi Du Wang, Cixi Da Bo Ge, Cixi City Club, Medical Ethics, Wang Baoqiang, Focus Report of CCTV, and others are actors with the highest intermediate centrality in the public opinion spreading network of the H7N9 incident. They have the most information and resources. They can communicate well with other actors and have the greatest influence on other actors. In the H7N9 sample network, there are not only a few in-charge actors with high intermediate centrality, but also actors with an intermediate centrality of 0. Among the 2369 actors involved, 1616 of them have an intermediate centrality of 0 and they cannot act as bridges. Indeed, they have almost no information and resources and are on the fringes of the network, the noninfluential, not to mention the ability to control information.

The article "Spread of Online Public Opinion of Animal Epidemic Emergency: A Case Study of the H7N9 Incident Based on Healthcare Data Analytics" was retracted in 2022. Reason: concerns about the peer review.

In public opinion spreading network of emergencies, the higher the intermediate central potential, the higher the likelihood that the information in the overall network is monopolized and controlled by a few people [16]. As shown in Table 2, the intermediate central potential of public opinion spreading network of the H7N9 incident was relatively high (45%), indicating that the public opinion spreading network of the H7N9 incident had a high connectivity and obvious bridging role, and some actors still had to obtain information through nodes with high intermediate central potential. The reason was that since the H7N9 animal epidemic emergency was related to the safety and security of the entire nation, the progress of the incident was usually released by the authority, and the netizens spread the public opinion through reposting, commenting, etc. Among them, Kaifu Lee, Wang Baoqiang, and other influential actors had their own influence and control over the spread of information resources. They can act as a bridge to enable the effective spread of relevant information.

### 3.5. Core-Periphery Analysis

As one of the methods to calculate agglomerated subgroups in terms of the frequency of relationships between actors, core-periphery analysis is suitable for identifying core group with higher density and peripheral group with lower density in the network [17]. The nodes in the core blocks are closely connected to each other, while the nodes in the peripheral blocks are sparsely connected to each other, and they all have the tendency to establish relationships with the core nodes [18]. The association model is shown as follows:

(4) $$\begin{array}{c} \rho =\sum_{i,j}\alpha_{ij}\delta_{ij},\;\delta_{ij}=\left\{\begin{array}{c} 1\\ 0 \end{array}\right.. \end{array}$$

Core-periphery analysis reflects the nature (core or periphery) of a specific node in the network. If *α*_*ij*_ = 1, there is a connection between nodes *i* and *j*; if *α*_*ij*_ = 0, there is no connection between nodes *i* and *j*. *C*_*i*_ reflects the nature (core or periphery) of node *i*. *δ*_*ij*_ represents the existence of an ideal state; only when *α*_*ij*_ = *δ*_*ij*_, the structure is a core-periphery structure, and the measure *ρ* at this time is at the maximum value, denoted by *ρ* (max).

Group 1 is the core actors in the public opinion spreading network of the H7N9 incident. It is composed of Toutiao News (Actor no. 1203), Xue Manzi (Actor no. 290), Xu Yongming (Actor no. 567), “Struggling in the secular” (Actor no. 676), “Interactive car-Li Nan” (Actor no. 1042), “gossip_ss” (Actor no. 19), “Bull eyes viewing of car” (Actor no. 41), “Ao Da Xia Nv” (Actor no. 105), “Forever Twenty-Two” (Actor no. 326), “Du Yi Si dUYi” (Actor no. 711), and other 15 members, which are in the center of the H7N9 opinion network and are closely connected to each other. Group 2 is composed of 2354 peripheral actors in the public opinion spreading network of the H7N9 incident, including “Beijing Cook” (Actor no. 775), “Freddie-Gemini” (Actor no. 1096), “Luo Bing” (Actor no. 106), “Da Gou Bang Guan Tian Xia” (Actor no. 107), “William_Wei Chao” (Actor no. 301), “Wu Gang” (Actor no. 336), “Qi Ran liya” (Actor no. 337), “Little_West” (Actor no. 477), “SFC_mushroom moon” (Actor no. 815), “SFC_mushroom moon” (Actor no. 941), “Ci Xi Du Wang” (Actor no. 1081), and “Feng Er Jiu” (Actor no. 1221). These nodes are basically unrelated and belong to a sparse group. The internal substructure results of spreading network of online public opinion of the H7N9 incident are shown in Table 4.

The article "Spread of Online Public Opinion of Animal Epidemic Emergency: A Case Study of the H7N9 Incident Based on Healthcare Data Analytics" was retracted in 2022. Reason: concerns about the peer review.

Toutiao News (Actor no. 1083) has reached the maximum core degree of 0.979 in the H7N9 opinion network, indicating that it is at the center of information resource exchange. It also has the greatest depth and breadth of information exchange with other actors. Then, the core degrees of MOP.com (Actor no. 553), Sina Video (Actor no. 40), Beijing Evening (Actor no. 1229), and Shanghai Morning Post (Actor no. 15) are 0.979, 0.124, 0.09, 0.07, and 0.068. These actors are key opinion leaders in the spreading of online public opinion of the H7N9 incident. The relevant information they publish, repost, or comment on Weibo is widely distributed and highly recognized.

### 3.6. Analysis of Out-In Degree

In a directed network, the point-centrality of a node is divided into in-degree and out-degree [19]. The number of times a node is reposting information from other nodes is called in-degree, which measures the breadth of the node's information sources. The number of times a node's information was reposted by other nodes is called out-degree, which measures the spread of the node's content in the network. The H7N9 incident public opinion network out-in degree measurement results are shown in Table 5.

As shown in Table 5, according to the measured out-degree and in-degree, the status of each node in the communication network and the richness of the information source can be measured. Actors such as Toutiao News, MOP.com, Sina Video, Beijing Evening, and DXY.cn are at the core of the network, and they are also important sources for other actors to follow and disseminate relevant public opinion information. Herein, Toutiao News (Actor no. 1083), MOP.com (Actor no. 2045), and Sina Video (Actor no. 1190) have the highest out-degree, which means that users tend to retweet relevant information posted by these users during spreading of online public opinion of the H7N9 incident. “Xue Manzi” (Actor no. 1378) and “Ji La-yamato-” (Actor no. 1366) has the richest sources of information, indicating that these nodes have the strongest interest in the spread of the event.

The article "Spread of Online Public Opinion of Animal Epidemic Emergency: A Case Study of the H7N9 Incident Based on Healthcare Data Analytics" was retracted in 2022. Reason: concerns about the peer review.

### 3.7. Analysis of Closeness Centrality

If the shortest path length between a node and other nodes is very short, then the closeness centrality of the node is high [20]. Absolute closeness centrality is calculated as (5) and relative closeness centrality as (6). The shortest distance between nodes *i* and *j* is represented by d_ij_, and *n* is the number of nodes. The H7N9 incident public opinion network closeness centrality measurement results are shown in Table 6.


(5) $$\begin{array}{c} C_{APi}^{-1}=\sum_{j=1}^{n}d_{ij}, \end{array}$$

(6) $$\begin{array}{c} C_{RPi}^{-1}=\frac{C_{APi}^{-1}}{n-1}, \end{array}$$

Farness and closeness reflect absolute and relative closeness centrality, respectively. The absolute closeness centrality of Toutiao News (Actor no. 1083) is the smallest in the network structure of H7N9 animal epidemic emergency, indicating that the total length of the shortest path from this node to other nodes in the network is the shortest. It is not easy to be controlled by other nodes, the information dissemination efficiency is high, and the spreading of information is faster. In order to accurately identify the most effective communicators in network, optimize available resources, and ensure effective spreading of network information, it should be included in the system of government interventions for online public opinion events. During public opinion spreading of animal epidemic emergency, appropriate monitoring and intervention should be implemented for actors with high closeness centrality such as Toutiao News, which can be relatively effective in early warning and control of information spreading process of animal epidemic emergency.

## 4. Conclusions

A complete summary of public opinion spreading network of this incident was carried out through the phase characteristics of the life cycle of public opinion spreading network of animal epidemic emergency and the structural characteristics of public opinion spreading network of the H7N9 incident. The following conclusions can be drawn:

1. The reason for the low completeness of the public opinion spreading network of the H7N9 incident is, on the one hand, the large size of network diagram due to large sample size (2369 nodes were involved). As the size of network diagram increases, the density of the overall network diagram is getting smaller. On the other hand, there is large percentage of peripheral actors. Peripheral actors exhibit low density as they have weak connection with other actors, and the interaction is almost zero. The H7N9 incident is a public health incident that affects the health of every citizen, with a high level of public participation, but low interaction, and more of a loose collective. During spreading of online public opinion of animal epidemic emergency, there will be a period of information explosion with strong output, that is, the explosion period. At this time, a large number of small groups with different cohesiveness are formed in the network, among which the oligarchic opinion groups, which are mainly composed of high authority media, have great influence, and are at the core of the network. The government should monitor the situation intensively and release reliable official information in time to dispel the anxiety of the public.
2. From the centrality of public opinion spreading of the H7N9 incident, well-known media users or celebrities, who combine popularity and authority, have shown the advantage of controlling information. Toutiao News, Shanghai Morning Post, Xie Na, Kaifu Lee, and other well-known users have shown different information dissemination influence and media information control in the public opinion spreading network; these actors are not easily controlled by other actors and will influence other actors during spreading of public opinion. For the same type of animal epidemics, in each stage of public opinion spreading, the government can introduce high authority and high credibility judicial or government official nodes at the center of the public opinion spreading network to enhance government-public interaction and establish effective communication channels with netizens. This behavior can be interpreted as “wave to ride.” For instance, by posting official messages under well-known media and celebrity users who commented on the incident, the government not only ensures accurate information is delivered but also achieves a soft control effect on governance. This method is especially good in the animal epidemic emergency stage. In the spreading stage of the information explosion, compulsory methods such as deleting posts and blocking IP can be used to control public opinion. In the fading phase, the clustering effect also fades, and the regulators can monitor the occurrence of related events at this time and try to avoid the occurrence of secondary negative public opinion.
3. The appropriate governance strategy for the different stages of public opinion is adopted. During the onset phase, animal epidemic emergency is characterized by dispersion, disorder, and instability. Taking advantage of this feature, animal epidemics related government nodes, such as China Health and Chinese Center for Disease Control and Prevention, should have the right to take the lead first, enhance their influence on the Internet, and make emergency plans in time according to the trend of public opinion. In the spreading stage, it is necessary to guide the information in an orderly manner in the massive explosion of information. Animal epidemic emergency presents the characteristics of hot topic, high concentration, and high output in this stage. These methods should be proactively applied to dispel people's doubts and dissatisfaction in a timely manner, so as to achieve effective interaction between government and the public, to understand and collect public opinion, to detect and clarify rumors early, to further weaken negative effects, and to prevent the recurrence of public opinion and the further spread of undesirable public opinion. In the fading phase, although the popularity is reduced and the topic is weakened, it cannot be taken lightly. The government should continue to monitor the incident. Especially in the case of animal epidemics, because the epidemic itself may be recurring and highly dangerous, it is very likely to trigger secondary public opinion or even multipeak public opinion, so it is extremely important to rebuild public credibility at this stage. The government and relevant authorities need to publicize government's active efforts, further preventive and curative measures, the development of vaccines, and tracking the recovery of patients. In addition, it is necessary to screen the Internet for content that is conductive to the formation of a healthy online culture, the healthy physical and mental development of Internet users, and the effective management of the government, to provide a good online environment that is conducive to the reestablishment of public confidence after the crisis.

The article "Spread of Online Public Opinion of Animal Epidemic Emergency: A Case Study of the H7N9 Incident Based on Healthcare Data Analytics" was retracted in 2022. Reason: concerns about the peer review.

## Figures and Tables

**Figure 1:** Life cycle of online public opinion of animal epidemic emergency.

**Figure 2:** The search index chart of keyword “H7N9” in Baidu Index.

**Figure 3:** Integrated spreading networks of online public opinion of the H7N9 incident.

**Table 1:** The three stages of spreading of public opinion of the H7N9 incident.

Stage	Dissemination characteristics and incident development
Occurrence stage 3.31–4.9 2013	The term H7N9 began to appear and quickly occupied the public's sight on March 31th, 2013. On the same day, there were three cases of H7N9 infection reported in Shanghai and Anhui Province. The Internet search index for “H7N9” also began to appear on March 31th and rose rapidly. On April 5, the National Health and Family Planning Commission began to release daily information on the H7N9 epidemic nationwide, and the search index for “H7N9” reached its first peak on that day. Because of the increased transparency and publicity of the information, public sentiment calmed down slightly [10]. From April 5th, the Chinese government website started to publish daily “information on the human H7N9 avian influenza epidemic,” which provided information on the number of confirmed cases of avian influenza, the distribution of areas, and the situation of infection and loss, and the authoritative information prevented the spread of rumors in time. Therefore, this paper defined the period from March 31th to April 9th as the stage of “H7N9” microblog public opinion occurrence. At this stage, public opinion spreading showed the characteristics of dispersion, disorder, and instability.
Spreading stage 4.10–4.12 2013	Along with the report of the first H7N9 patient being cured on April 10th, the online attention of the H7N9 incident surged, pushing the incident to the outbreak of public opinion. After April 11th, the H7N9 incident showed a downward trend, and online public opinion gradually dropped. Therefore, April 10–12th was determined as the spreading stage of the “H7N9” microblog. At this stage, public opinion spreading showed the characteristics of high popularity, high concentration, and high output.
Fading stage 4.13–4.25 2013	The country followed up on the epidemic information, which was released on a daily basis. Cases across the country were sporadic. Every region was focusing on treatment and prevention. The epidemic started to be effectively alleviated and controlled. On April 16th, a total of 78 human cases of H7N9 avian influenza were confirmed nationwide, with 16 deaths [11]. Starting from April 25th, the frequency of the National Health and Family Planning Commission's epidemic release was changed to once every 5 days, and the number of new cases decreased and the outbreak was basically under control. The number of new cases was reduced and the epidemic was basically under control. Correspondingly, the discussion of H7N9 among Internet users gradually faded. Therefore, April 13th–April 25th was identified as the fading phase of the H7N9 incident public opinion. At this stage, the outbreak was basically under control.

**Table 2:** Measured network density of spreading of online public opinion of the H7N9 incident.

Network density (density)	Number of interaction connection ties (no. Of ties)
0.0005	3178

**Table 3:** Measured intermediate centrality of public opinion spreading network of the H7N9 incident (first 30).

No.	ID	Intermediate centrality	No.	ID	Intermediate centrality
1083	Toutiao News	25204	2306	Wa Yu	392
603	a1400273289	17412	2345	Kai Xin Guo jll	376
359	Kaifu Lee	15618	2355	Liu Heting is a big fool who loves 2PM	360
1500	Changzhou Daily News Tongtong	3901	2359	Hu Ting kt	344
331	Luo Yonghao Smartisan handphone	3901	560	Yi ye zhi qiu	330
2045	MOP.com	2963	2361	Wo ma lei di ga ga-JY	328
1959	Cixi Du Wang	2835	432	YU-Fion	315
1929	Cixi Da Bo Ge	2333	2363	Rou Rou Xiao Xiao Wo	312
1845	Cixi City Club	2324	367	So_____________________	300
1664	Medical Ethics	1962	2365	Mini_minijiji	296
429	Wang Baoqiang	1962	312	Magger X Gao Gao	285
447	Focus Report of CCTV	1960.5	2367	Chen Yan 1115	280
438	Lin Zai-_-	1960.5	277	Ruby Wen	270
1378	Xue Manzi	418	1996	Xing fu Le le qing	270
2220	Lu_Sheng_	408	1810	Song Qian-fx--victoria	266

Network Centralization index = 45%.

The article "Spread of Online Public Opinion of Animal Epidemic Emergency: A Case Study of the H7N9 Incident Based on Healthcare Data Analytics" was retracted in 2022. Reason: concerns about the peer review.

**Table 4:** Core-periphery analysis results of spreading network of online public opinion of the H7N9 incident (first 30).

No.	ID	Core degree	No.	ID	Core degree
1203	Toutiao News	0.979	301	William_Wei Chao	0.006
553	MOP.com	0.124	336	Wu Gang	0.006
40	Sina Video	0.09	337	Qi ran liya	0.006
1229	Beijing Evening	0.07	477	Little_West	0.006
15	Shanghai Morning Post	0.068	815	SFC_mushroom moon	0.006
290	Xue Manzi	0.028	941	Si Yang Yan Hao	0.006
1376	Lao Chen	0.026	1081	Ci Xi Du Wang	0.006
512	DXY.cn	0.015	1221	Feng Er Jiu	0.006
696	Hot topics in Weibo	0.013	1258	Xiao Xin_Xia Yi Wei Qing	0.006
996	nownow	0.013	1359	Trouble_AQ	0.006
424	Cixi City Club	0.009	1363	Singapore Shangrila-Herb	0.006
775	Beijing Cook	0.009	1392	Nue Yang Kuang Ren Shou Sheng Xia Ying	0.006
1096	Freddie-Gemini	0.009	1415	Sincere Liu	0.006
106	Luo Bing	0.006	20	You should call me Meng Da Da Da Da Da Ren	0.004
107	Da Gou Bang Guan Tian Xia	0.006	61	Xiao Xun'er Jiu Shi Ye Zhi	0.004

**Table 5:** Out-in degree of spreading of online public opinion of the H7N9 incident (partial).

No.	ID	Out-degree	In-degree	No.	ID	Out-degree	In-degree
1083	Toutiao News	689	2	1752	Beijing Cook	4	1
2045	MOP.com	91	1	1680	SFC_mushroom moon	3	1
1190	Sina Video	61	0	1366	Ji La-yamato-	3	3
1986	Shanghai Morning Post	55	0	481	SFC Luo Jia Xiao Wen	3	1
1852	Beijing Evening	49	0	427	Xiao Xi_Xia Yi Wei Qing	3	1
1378	Xue Manzi	20	3	521	Da Gou Bang Guan Tian Xia	3	2
1683	Lao Chen	13	1	2316	William_Weichao	3	2
1973	DXY.cn	12	2	486	Deng Meng Meng Catch Er Jing Jing	3	1
1908	nownow	8	2	1982	Si Ma Ping Bang	3	1
1222	Hot topics in Weibo	7	1	1820	Pi Ren Ri Ji	3	2
1845	Cixi City Club	4	1	1358	Luo Bing	3	2
1419	Qiyan liya	4	3	1951	Mao Ku Sang Mookoo	3	1
900	Wu Gang	4	1	1544	Feng Er Jiu	3	3
822	Freddie-Gemini	4	1	436	RP Cun Mang Ni Qiu 2013Yi Qie Shun Li de Bao	3	2
738	Interactive cars-Li Nan	4	2	918	Si Yang Yang Hao	3	2

The article "Spread of Online Public Opinion of Animal Epidemic Emergency: A Case Study of the H7N9 Incident Based on Healthcare Data Analytics" was retracted in 2022. Reason: concerns about the peer review.

**Table 6:** Closeness centrality of online public opinion of the H7N9 incident (partial).

No.	ID	Farness	Closeness	No.	ID	Farness	Closeness
1083	Toutiao News	18421	12.855	805	Annie Wang Xinyi	34864	6.792
1986	Shanghai Morning Post	20125	11.766	2311	KDS Broadband	38839	6.097
1849	Ying Mu Hua Dao	20224	11.709	2311	KDS Broadband	38839	6.097
1378	Xue Manzi	20303	11.663	2303	Single tone	38840	6.097
302	Xie Na	23085	10.258	2318	C2-KGB Gun Angel	38840	6.097
359	Kaifu Lee	23091	10.255	2364	1988_Jing	39475	5.999
1224	FYVVM	23095	10.253	2363	Rou Rou Xiao Xiao Wo	39475	5.999
1923	Jia Xiaoyu-Yoyiki	23104	10.249	33	Communist Youth League Committee of Xinxiang	39493	5.996
1857	Xiahe	24089	9.83	18	Wang Weiming	39493	5.996
2162	Chen He	24250	9.765	2298	Jiuting Community Network	41197	5.748
179	He Jiong	25411	9.319	2307	Hot Spots in Shanghai Today	41195	5.748
195	Jiaxing Grassroots News	25486	9.291	1715	Tianjin Mo	48947	4.838
2191	Shanghai Songjiang Forum	27093	8.74	203	Zhang Normal University Work center	600322	0.042
90	Xiao Q Ye Wei Bo	27823	8.511	121	Smelly blog	600323	0.042
2266	Guangzhou Police	30201	7.841	190	Min Normal University 11	600323	0.042

## Data Availability

Data sharing is not applicable to this article as no datasets were generated or analyzed during the current study.
